The article "Correlation between hs-CRP, IL-6, IL-10, ET-1, and Chronic Obstructive Pulmonary Disease Combined with Pulmonary Hypertension" was published in 2022. Journal: J Healthc Eng.

# Correlation between hs-CRP, IL-6, IL-10, ET-1, and Chronic Obstructive Pulmonary Disease Combined with Pulmonary Hypertension

**DOI:** 10.1155/2022/3247807

**Published:** 2022-02-10

**Authors:** Danfen Yang, Li Wang, Pengfei Jiang, Rui Kang, Yuanyuan Xie

**Affiliations:** ^1^Department of Geriatrics, Affiliated Hospital of Yan'an University, Yan'an 716000, Shaanxi, China; ^2^Department of Respiratory, Affiliated Hospital of Yan'an University, Yan'an 716000, Shaanxi, China; ^3^Department of Orthopedics, Affiliated Hospital of Yan'an University, Yan'an 716000, Shaanxi, China

## Abstract

With the development of society, chronic obstructive pulmonary disease (COPD), a common respiratory disease, suffers an increasing incidence. To explore the correlation between high-sensitivity C-reactive protein (hs-CRP), interleukin-6 (IL-6), interleukin-10 (IL-10), endothelin-1 (ET-1), and chronic obstructive pulmonary disease combined with pulmonary hypertension (COPD-PH), a total of 112 COPD patients admitted to our hospital from July 2017 to December 2020 were analyzed prospectively, of which 57 patients combined with PH were enrolled in the research group and the other 55 patients without PH were enrolled in the control group. Serum hs-CRP, IL-6, IL-10, ET-1, blood gas indexes, and related indexes of lung function of the two groups were detected and their correlations were analyzed. The research group was divided into the mild group, moderate group, and heavy group according to pulmonary average arterial pressure, and serum hs-CRP, IL-6, IL-10, ET-1, and disease severity were analyzed. Receiver operating characteristic curve (ROC) analysis was performed to serum hs-CRP, IL-6, IL-10, and ET-1 of COPD-PH patients, and independent risk factors for COPD-PH were analyzed. The research group showed significantly higher serum hs-CRP, IL-6, and ET-1 and significantly lower IL-10 expression than the control group (all *P* < 0.05); serum hs-CRP, IL-6, and ET-1 were negatively correlated with PaO2, FEV1, FVC, and FEV1/FVC and positively correlated with PaCO2; IL-10 was positively correlated with PaO2, FEV1, FVC, and FEV1/FVC and negatively correlated with PaCO2; hs-CRP, IL-6, and ET-1 were positively correlated with COPD-PH severity, and IL-10 was negatively correlated with it. hs-CRP, IL-6, IL-10, and ET-1 were closely and significantly related to the pathological process of COPD-PH, including onset and development, and the elevation of hs-CRP, IL-6, and ET-1 and decrease of IL-10 are independent risk factors for the onset of COPD-PH. With relatively high predictive value for COPD-PH, hs-CRP, IL-6, IL-10, and ET-1 can be promoted as predictors for it.

## 1. Introduction

With the development of society, chronic obstructive pulmonary disease (COPD), a common respiratory disease, suffers an increasing incidence [1]. Pulmonary hypertension (PH), one of the main complications of COPD, is a disease for pulmonary vascular endothelial function disorder and pulmonary vascular remodeling due to hypoxic pulmonary vasoconstriction for repeated acute disease exacerbation of patients, and it is also one of the important factors leading to poor prognosis of COPD patients [2, 3]. A study for secondary PH indicated that systemic inflammation and hypoxia play an important role in the pathogenesis of PH [4].

In recent years, the role of inflammatory response in the secondary PH of COPD has drawn much attention, and it is believed that a variety of inflammatory factors play an important role in the regulation of pulmonary artery pressure [5, 6]. High-sensitivity C-reactive protein (hs-CRP) is an acute reactive protein synthesized by the liver. A study pointed out that hs-CRP is an important index of systemic inflammatory response, and its expression level will not be affected by cortical hormone treatment [7]. As relatively representative inflammatory factors, interleukin-6 (IL-6) and interleukin-10 (IL-10) also play an important role in the pathogenesis of PH [8]. Endothelin is a factor proven to be with an important function in pulmonary vascular resistance increase and pulmonary vascular remodeling, and endothelin-1 (ET-1) is one of the most important factors of it [9]. PH is a disease characterized by progressive rising of pulmonary vascular resistance. When COPD causes airway obstruction and damages pulmonary parenchyma and pulmonary vasculature, pulmonary arterial endothelium will suffer hyperplasia and fibrosis, eventually leading to pulmonary circulation remodeling and onset of PH. A study pointed out that ET-1 expression has a very close relationship with the degree of distal pulmonary vascular damage [10]. This study aims to explore the correlation between high-sensitivity C-reactive protein (hs-CRP), interleukin-6 (IL-6), interleukin-10 (IL-10), endothelin-1 (ET-1), and chronic obstructive pulmonary disease combined with pulmonary hypertension (COPD-PH).

Therefore, this study explored the correlation between hs-CRP, IL-6, IL-10, ET-1, and COPD-PH, so as to provide a more theoretical basis for early intervention and treatment for COPD-PH patients.

## 2. Materials and Methods

### 2.1. General Materials

A total of 112 COPD patients (65.21 ± 4.77 years old in mean age) admitted to our hospital from July 2015 to December 2018 were analyzed prospectively, of which 57 patients combined with PH were enrolled in the research group and other 55 patients without PH were enrolled in the control group. Inclusion criteria: patients meeting the diagnostic criteria for COPD and patients (to be enrolled in the research group) meeting the diagnostic criteria in 2009 European Pulmonary Hypertension Guidelines. Exclusion criteria: patients with other complications, primary diseases of lungs, severe hepatic renal dysfunction, other malignant tumors or severe immune system disease, patients with communication obstacles and cognitive impairment, and patients unwilling to cooperate for the experiment. The experiment has been approved by the ethics committee of our hospital, and all patients and their families agreed to participate in the experiment and signed an informed consent form.

### 2.2. Related Index Detection

#### 2.2.1. Blood Gas Index and Related Inflammatory Factor Detection

Blood gas analysis was performed on all patients after admission (determined by an ABL700 blood gas analyzer from Danish Radiometer Medical Equipment Co., Ltd.), and 5 ml of fasting venous blood taken in the next morning after admission was centrifuged at 3000 r/min and stored at −80°C for later detection. hs-CRP was determined by an automatic biochemistry analyzer through immune turbidimetry, and IL-6, IL-10, and ET-1 were determined by ELISA (IL-6 and IL-10 ELISA kits were purchased from Shanghai Jining Industrial Biotechnology Co., Ltd., N110863, N110820; ET-1 kit was purchased from Beijing Reanta Biotechnology Co., Ltd., YAD) in strict accordance with kit instructions.

#### 2.2.2. Pulmonary Function Detection

Pulmonary function indexes were detected for all patients after admission based on the premise that the patients have not received bronchodilator or glucocorticoid drugs within 48 hours before pulmonary function detection, which mainly included the detection and calculation of forced expiratory volume in one second (FEV1), forced vital capacity (FVC), and FEV1/FVC of patients.

#### 2.2.3. Pulmonary Artery Pressure Determination

All patients were determined in pulmonary artery pressure through a color doppler echocardiography in a peaceful supine position, and the four chamber images of their apical muscular were taken based on the premises of keeping sample lines parallel to regurgitation. The patients' PH was calculated according to the Bernoulli simplified formula: PASP = 4V2 (maximum tricuspid regurgitation rate) + 5 mmHg [11].

#### 2.2.4. Statistical Analysis

In the study, SPSS 19.0 software (Bizinsight (Beijing) Information Technology Co., Ltd.) was adopted for statistical analysis of experiment data; count data were analyzed by the chi-square test, and measurement data were expressed in mean ± standard deviation. Comparison between the two groups was tested by *t*, and their correlations were analyzed using the Pearson correlation coefficient. Logistic multivariate analysis was performed for risk factors of PH. *P* < 0.05 indicated statistical difference.

## 3. Results

### 3.1. Comparison in General Materials

There were no significant differences in gender, age, and body mass index (BMI) between the two groups (all *P* > 0.05). More details are given in Table 1.

### 3.2. Comparison between the Two Groups in Serum hs-CRP, IL-6, IL-10, and ET-1 Expression

The research group showed significantly higher serum hs-CRP, IL-6, and ET-1 and significantly lower IL-10 expression than the control group (all *P* < 0.05). More details are given in Table 2.

### 3.3. Related Blood Gas Index Detection of the Two Groups

In terms of blood gas index, the research group showed significantly lower PaO2 and significantly higher PaCO2 than the control group (both *P* < 0.05). More details are given in Table 3.

### 3.4. Pulmonary Function Indexes and Pulmonary Average Arterial Pressure of the Two Groups

The research group showed significantly lower FEV1, FVC, and FEV1/FVC and significantly higher pulmonary average arterial pressure than the control group (all *P* < 0.05). More details are given in Table 4.

### 3.5. Correlation Analysis of Serum hs-CRP, IL-6, IL-10, ET-1, and Blood Gas Indexes

Serum hs-CRP, IL-6, and ET-1 were negatively correlated with PaO2 (*P* < 0.001) and positively correlated with PaCO2 (*P* < 0.001). IL-10 was positively correlated with PaO2 (*P* < 0.001) and negatively correlated with PaCO2 (*P* < 0.001). More details are given in Table 5 and Figure 1.

### 3.6. Correlation Analysis of Serum hs-CRP, IL-6, IL-10, ET-1, and Pulmonary Function Indexes

Serum hs-CRP, IL-6, and ET-1 were negatively correlated with FEV1, FVC, and FEV1/FVC (all *P* < 0.05), and ET-1 was positively correlated with FEV1, FVC, and FEV1/FVC (all *P* < 0.05). More details are given in Table 6 and Figure 2.

### 3.7. Correlation Analysis of Serum hs-CRP, IL-6, IL-10, ET-1, and Severity of COPD

According to pulmonary average arterial pressure, the patients were divided into the mild group (40–50 mmHg, 17 patients), moderate group (50–65 mmHg, 24 patients), and heavy group (>65 mmHg, 16 patients). Comparison showed that the more severe the patients' disease, the higher the patients' hs-CRP, IL-6, and ET-1 expression and the lower the IL-10 expression. The correlation was statistically significant (*P* < 0.05). More details are given in Table 7. In addition, correlation analysis showed that the severity of the disease was positively correlated with hs-CRP, IL-6, and ET-1 (*r* = 0.808, *P* < 0.05; *r* = 0.883, *P* < 0.03; *r* = 0.817, *P* < 0.05) and negatively correlated with IL-1 (*r* = −0.597, *P* < 0.05). More details are shown in Figure 3.

### 3.8. ROC Analysis of hs-CRP, IL-6, IL-10, and ET-1 to COPD-PH

In terms of COPD-PH diagnosis, hs-CRP showed sensitivity of 90.91%, specificity of 85.96%, area-under-the-curve (AUG) of 0.899, and critical value of 38.49 (mg/L); IL-6 showed sensitivity of 87.27%, specificity of 89.47%, AUG of 0.929, and critical value of 98.99 (pg/mL); IL-10 showed sensitivity of 81.82%, specificity of 68.42%, AUG of 0.854, and critical value of 4.740 (pg/mL), and ET-1 showed sensitivity of 87.27%, specificity of 57.89%, AUG of 0.805, and critical value of 39.64 (pg/mL). More details are shown in Figure 4.

### 3.9. Multivariate Analysis of the Incidence of PH

The above study indicated that elevation of hs-CRP, IL-6, and ET-1 and decrease of IL-10 were correlated with COPD-PH. Assignment was done to those factors (Table 8), and logistic regression analysis was performed to analyze whether those factors were independent risk factors for the onset of COPD-PH, and it turned out that elevation of hs-CRP (OR: 2.314, 95% CI: 1.104–4.211), IL-6 (OR: 2.564, 95% CI: 1.114–4.789), and ET-1 (OR: 3.759, 95% CI: 1.229–5.116) and decrease of IL-10 (OR: 6.151, 95% CI: 3.119–5.243) were all independent risk factors for the onset of COPD-PH. More details are given in Table 9.

## 4. Discussion

COPD is a respiratory disease characterized by restricted flow and damaged lung tissue [12]. PH is a disease characterized by the progressive rising of pulmonary vascular resistance. When COPD causes airway obstruction and damages pulmonary parenchyma and pulmonary vasculature, pulmonary arterial endothelium will suffer hyperplasia and fibrosis, eventually leading to pulmonary circulation remodeling and the onset of PH [13, 14]. PH in COPD patients is an irreversible pathological change, which has an important impact on the patient's poor prognosis [15].

A study pointed out that the incidence of COPD-PH is closely related to the inflammatory response [16], so the study explored the expression of several representative inflammatory factors of COPD-PH and their correlation with it. First, the two groups were compared in hs-CRP, IL-6, IL-10, and ET-1 expression, and it turned out that the research group showed significantly higher serum hs-CRP, IL-6, and ET-1 and significantly lower IL-10 expression than the control group, which indicated that COPD patients with PH and COPD patients without PH showed a significant difference in hs-CRP, IL-6, IL-10, and ET-1 expression and further suggested that the onset of COPD is related to systemic inflammatory response. hs-CRP, a typical sensitivity index of low-level inflammatory state produced by liver epithelial cells for stimulation by IL-6 and other factors, can stimulate the release of inflammatory mediators such as ET-1 and further expand inflammatory response [17, 18]. A study pointed out that ET-1, the most potent vasoconstrictor ever discovered, can promote lung vascular endothelium hyperplasia and fibrosis and aggravate pulmonary artery remodeling [19]. IL-6, a multifunctional proinflammatory cytokine, plays a key role in the development of inflammatory response [20]. A study about hypoxia inducible mice pointed out that IL-6 involved in pulmonary inflammation and pulmonary vascular remodeling of mice and believed that L-6 involved in the effects of PH [21]. IL-10 is an anti-inflammatory factor that can inhibit the expansion of inflammatory response. A study pointed out that COPD-PH patients have significantly lower serum IL-10 than the patients with COPD alone [22]. In addition, a study pointed out that increased pulmonary artery mechanical pressure will damage vascular endothelial cells, promote the release of inflammatory factors such as IL-6, and cause the liver to release hs-CRP through synthesis [23]. All of the above studies have confirmed and explained our experimental results.

In order to further explore the correlation between hs-CRP, IL-6, IL-10, ET-1, and PH, blood gas indexes and related indexes of lung function of the two groups were detected, and their correlations have been analyzed, and it turned out that serum hs-CRP, IL-6, and ET-1 were negatively correlated with PaO2, FEV1, FVC, and FEV1/FVC and positively related to PaCO2. It may be due to the fact that inflammatory factors are involved in PH formation, and the formation will further lead to an increase in blood inflammatory factors of patients, causing a vicious circle. IL-10 was positively related to PaO2, FEV1, FVC, and FEV1/FVC and negatively elated to PaCO2. In addition, the correlation of serum hs-CRP, IL-6, IL-10, ET-1, and COPD-PH severity was analyzed, and it turned out that hs-CRP, IL-6, and ET-1 were positively correlated with COPD-PH severity, and IL-10 was negatively correlated with COPD-PH severity, which indicated that serum hs-CRP, IL-6, IL-10, and ET-1 were closely related to the severity of the disease and may be used as predictors for the disease.

In order to further analyze the influence of hs-CRP, IL-6, IL-10, and ET-1 on COPD-PH patients, ROC analysis was performed, and the results indicated that hs-CRP, IL-6, IL-10, and ET-1 have relatively high predictive value for COPD-PH. Then, assignment was performed to critical values, and logistic regression analysis was carried out. It indicated that elevation of hs-CRP, IL-6, and ET-1 and decrease of IL-10 were all independent risk factors for the onset of COPD-PH. It further suggested that inflammatory factors including hs-CRP, IL-6, IL-10, and ET-1 play important roles in the onset and progression of COPD-PH. A study about the influence of inflammatory factors on COPD-PH pointed out that IL-6 and CRP may be independent risk factors for COPD-PH, which is consistent with some of our results [24]. Direct determination of PH in COPD is traumatic, so it is of great clinical significance to detect hs-CRP, IL-6, IL-10, and ET-1 to monitor pulmonary hypertension [25].

## 5. Conclusion

In conclusion, hs-CRP, IL-6, IL-10, and ET-1 were closely and significantly related to the pathological process of COPD-PH, including onset and development, and the elevation of hs-CRP, IL-6, and ET-1 and decrease of IL-10 are independent risk factors for the onset of COPD-PH. With relatively high predictive value for COPD-PH, hs-CRP, IL-6, IL-10, and ET-1 can be promoted as predictors for it. There are certain shortcomings of this study. For example, the diagnostic value of hs-CRP, IL-6, IL-10, and ET-1 for COPD-PH severity was not explored, and because of limited number of samples included, the conclusion may be exploratory. In the subsequent research, we will include more samples and supplement the details of the experiment to make the conclusion more substantial.

## Figures and Tables

**Figure 1:** Correlation analysis of serum hs-CRP, IL-6, IL-10, ET-1, and blood gas indexes. (a) Negative correlation between hs-CRP and PaO2 (*r* = −0.776, *P* < 0.001). (b) Positive correlation between hs-CRP and PaCO2 (*r* = 0.780, *P* < 0.001). (c) Negative correlation between IL-6 and PaO2 (*r* = −0.786, *P* < 0.001). (d) Positive correlation between IL-6 and PaCO2 (*r* = 0.871, *P* < 0.001). (e) Positive correlation between IL-10 and PaO2 (*r* = 0.594, *P* < 0.001). (f) Negative correlation between IL-10 and PaO2 (*r* = −0.709, *P* < 0.001). (g) Negative correlation between ET-1 and PaO2 (*r* = −0.709, *P* < 0.001). (h) Positive correlation between ET-1 and PaCO2 (*r* = 0.797, *P* < 0.001).

**Figure 2:** Correlation analysis of serum hs-CRP, IL-6, IL-10, ET-1, and pulmonary function indexes. (a) Negative correlation between hs-CRP and FEV1 (*r* = −0.725, *P* < 0.001). (b) Negative correlation between hs-CRP and FVC (*r* = −0.759, *P* < 0.001). (c) Negative correlation between hs-CRP and FEV1/FVC (*r* = −0.808, *P* < 0.001). (d) Negative correlation between IL-6 and FEV1 (*r* = −0.783, *P* < 0.001). (e) Negative correlation between IL-6 and FVC (*r* = −0.835, *P* < 0.001). (f) Negative correlation between IL-6 and FEV1/FVC (*r* = −0.811, *P* < 0.001). (g) Positive correlation between IL-10 and FEV1 (*r* = 0.520, *P* < 0.001). (h) Positive correlation between IL-10 and FVC (*r* = 0.601, *P* < 0.001). (i) Positive correlation between IL-10 and FEV1/FVC (*r* = 0.580, *P* < 0.001). (j) Negative correlation between ET-1 and FEV1 (*r* = −0.816, *P* < 0.001). (k) Negative correlation between ET-1 and FVC (*r* = −0.785, *P* < 0.001). (l) Negative correlation between ET-1 and FEV1/FVC (*r* = −0.701, *P* < 0.001).

**Figure 3:** Correlation analysis of hs-CRP, IL-6, IL-10, ET-1, and COPD-PH severity. (a) Positive correlation between hs-CRP and severity of the disease (*r* = 0.808, *P* < 0.05). (b) Positive correlation between IL-6 and severity of the disease (*r* = 0.883, *P* < 0.03). (c) Negative correlation between IL-10 expression and severity of the disease (*r* = −0.597, *P* < 0.05). (d) Positive correlation between ET-1 and severity of the disease (*r* = 0.817, *P* < 0.05).

**Figure 4:** ROC analysis of hs-CRP, IL-6, IL-10, and ET-1 to COPD-PH. In terms of COPD-PH diagnosis, (a) hs-CRP shows sensitivity of 90.91%, specificity of 85.96%, AUG of 0.899, and critical value of 38.49 (mg/L); (b) IL-6 shows sensitivity of 87.27%, specificity of 89.47%, AUG of 0.929, and critical value of 98.99 (pg/mL); (c) IL-10 shows sensitivity of 81.82%, specificity of 68.42%, AUG of 0.854, and critical value of 4.740 (pg/mL); (d) ET-1 shows sensitivity of 87.27%, specificity of 57.89%, AUG of 0.805, and critical value of 39.64 (umol/L).

**Table 1:** General condition (*n* (%)).

Factor	The research group, *n* = 57	The control group, *n* = 55	*t*/*χ*^2^	*P*
Gender			0.002	0.964
Male	35 (61.40)	34 (61.82)		
Female	22 (38.60)	21 (38.18)		
Age (Y)			0.001	0.975
≤65	24 (42.10)	23 (41.82)		
>65	33 (57.90)	32 (58.18)		
BMI (kg/m^2^)			0.000	0.992
≤22	27 (47.37)	26 (47.27)		
>22	30 (52.63)	29 (52.73)		
Smoking history			0.007	0.932
Yes	40 (70.18)	39 (70.91)		
No	17 (29.82)	16 (29.09)		
Course of disease	4.31 ± 2.21	4.29 ± 2.19	0.049	0.961
Coagulation function				
APTTs	27.91 ± 2.02	28.05 ± 2.04	0.368	0.713
PTs	11.54 ± 1.23	11.57 ± 1.21	0.131	0.896
FIB g/l	3.15 ± 0.14	3.16 ± 0.13	0.395	0.694
Education level				
With junior high school diploma and below	29 (50.88)	28 (50.91)	0.000	0.997
With junior high school diploma and above	28 (49.12)	27 (49.09)		

**Table 2:** Comparison between the two groups in serum hs-CRP, IL-6, IL-10, and ET-1 expression.

Factor	The research group, *n* = 57	The control group, *n* = 55	*t*	*P*
hs-CRP (mg/L)	42.76 ± 3.54	37.27 ± 1.37	10.75	<0.001
IL-6 (pg/mL)	104.68 ± 8.35	93.12 ± 6.32	8.239	<0.001
IL-10 (pg/mL)	4.38 ± 0.45	5.23 ± 0.37	10.90	<0.001
ET-1 (umol/L)	43.91 ± 9.94	30.18 ± 7.59	8.195	<0.001

**Table 3:** Related blood gas index detection of the two groups.

Factor	The research group, *n* = 57	The control group, *n* = 55	*t*	*P*
PaO2 (mmHg)	69.26 ± 8.19	95.19 ± 10.65	14.47	<0.001
PaCO2 (mmHg)	56.39 ± 9.28	43.19 ± 7.56	8.236	<0.001

**Table 4:** Pulmonary function indexes and pulmonary average arterial pressure of the two groups.

Factor	The research group, *n* = 57	The control group, *n* = 55	*t*	*P*
FEV1 (%)	50.98 ± 4.18	64.51 ± 5.39	14.88	<0.001
FVC (%)	63.71 ± 4.26	72.23 ± 6.51	8.224	<0.001
FEV1/FVC	51.19 ± 5.54	57.71 ± 6.37	5.786	<0.001
Pulmonary average arterial pressure (mmHg)	59.61 ± 15.35	24.19 ± 5.47	34.64	<0.001

**Table 5:** Correlation analysis of serum hs-CRP, IL-6, IL-10, ET-1, and blood gas indexes.

Index	PaO2		PaCO2	
	*r*	*P*	*r*	*P*
hs-CRP	−0.776	<0.001	0.780	<0001
IL-6	−0.786	<0.001	0.871	<0.001
IL-10	0.594	<0.001	−0.617	<0.001
ET-1	−0.709	<0.001	0.797	<0.001

**Table 6:** Correlation analysis of serum hs-CRP, IL-6, IL-10, ET-1, and pulmonary function indexes.

Index	FEV1		FVC		FEV1/FVC	
	*r*	*P*	*r*	*P*	*r*	*P*
hs-CRP	−0.725	<0.001	−0.759	<0.001	−0.808	<0.001
IL-6	−0.783	<0.001	−0.835	<0.001	−0.811	<0.001
IL-10	0.520	<0.001	0.601	<0.001	0.580	<0.001
ET-1	−0.816	<0.001	−0.785	<0.001	−0.701	<0.001

**Table 7:** Blood gases hs-CRP, IL-6, IL-10, and ET-1 expression in patients with different severities of disease in the research group.

Factor	The mild group, *n* = 17	The moderate group, *n* = 24	The heavy group, *n* = 16	*F*	*P*
hs-CRP (mg/L)	38.51 ± 1.01	42.76 ± 2.19	45.76 ± 3.54	37.83	<0.001
IL-6 (pg/mL)	99.29 ± 5.13	105.11 ± 6.13	109.91 ± 7.19	17.15	<0.001
IL-10 (pg/mL)	4.88 ± 0.45	4.43 ± 0.43	3.92 ± 0.41	20.49	<0.001
ET-1 (umol/L)	40.16 ± 5.21	44.81 ± 6.33	49.26 ± 7.19	8.657	<0.001

**Table 8:** Assignment.

Items	Assignment
hs-CRP	≤38.49 (mg/L) = 1, >38.49 (mg/L) = 2
IL-6	≤98.99 (pg/mL) = 1, >98.99 (pg/mL) = 2
IL-10	≤4.740 (pg/mL) = 1, >4.740 (pg/mL) = 2
ET-1	≤39.64 (umol/L) = 1, >39.64 (umol/L) = 2

**Table 9:** Multivariate analysis.

Factors	*β*	S.E	Wald	OR	95% CI	*P*
hs-CRP	2.793	0.425	1.983	2.314	1.104–4.211	<0.01
IL-6	3.149	0.613	2.197	2.564	1.114–4.789	<0.01
IL-10	3.169	0.642	2.231	6.151	3.119–5.243	<0.01
ET-1	3.496	0.741	2.621	3.759	1.229–5.116	<0.01

## Data Availability

The datasets used and/or analyzed during the current study are available from the corresponding author upon request.
